# *Citrus maxima* (Brum.) Merr. (Rutaceae): Bioactive Chemical Constituents and Pharmacological Activities

**DOI:** 10.1155/2022/8741669

**Published:** 2022-05-30

**Authors:** Biswash Sapkota, Hari Prasad Devkota, Prakash Poudel

**Affiliations:** ^1^Department of Pharmacy, Madan Bhandari Academy of Health Sciences, Hetauda 44100, Nepal; ^2^Graduate School of Pharmaceutical Sciences, Kumamoto University, 5-1 Oe-honmachi, Chuo-ku, Kumamoto 862-0973, Japan; ^3^Pharmacy Program, Gandaki University, Pokhara 33700, Nepal

## Abstract

*Citrus maxima* (Burm). Merr. (family Rutaceae), commonly known as Pomelo, is an ethnomedicinally, pharmacologically, and phytochemically valued species. Various ethnomedicinal reports have revealed the use of *C. maxima* for cough, fever, asthma, diarrhea, ulcer, and diabetes and as a sedative. Numerous phytochemicals have been reported from *C. maxima* such as polyphenols, terpenoids, sterols, carotenoids, vitamins, and amino acids. The plant possesses significant bioactivities like antioxidant, antimicrobial, anti-inflammatory, analgesic, anticancer, antidiabetic, anti-Alzheimer's disease, insecticidal, anxiolytic, hepatoprotective, antimalarial, and antiobesity. Extensive research is necessary to explore the detailed mechanism of action of extracts and compounds to design effective medicines, herbal products, and functional foods.

## 1. Introduction

*Citrus maxima* (Burm). Merr. (syn. *Citrus grandis* (L.) Osbeck) (Figure 1) belongs to the family Rutaceae. It is a perennial tree commonly known as Pomelo, Bhogate, Shaddock, Papanus, Pummelo, etc. in various parts of the world, as shown in Table 1. The plant is indigenous to Asia and is commercially grown in China, Nepal, Thailand, Malaysia, India, Vietnam, Indonesia, Philippines, Japan, and many other Asian countries. Lately, it has been introduced to many tropical nations [1–3]. It grows widely in temperatures 25–32°C and rainfall 1,500–2,500 mm within a 3-4 months dry season. It raises well in rough sand to heavy clay but favors fertile soils [2, 3]. Figure 1 shows various plant parts of *C. maxima,* which include the whole plant, whole fruit, albedo, and pulp. It has big round-shaped edible fruits with pink or white flesh. It is traditionally used for ulcers, febrifuge, dyspepsia, lumbago, fever, cardiotonic, gastrointestinal disorders, diabetes, and cardiovascular disease [4–9]. Various chemical constituents are reported from many parts of the *C. maxima* plant. The extracts or pure compounds from this plant have also been evaluated for a wide range of biological activities. The aim of this review article is to provide comprehensive outline of phytochemistry and pharmacological aspects of the plant and to attract scientific communities for further studies on possible utilization of *C. maxima* in the field of pharmaceutical, nutraceutical, and cosmeceutical industry.

## 2. Methodology

Scientific information about ethnomedicinal uses, phytoconstituents, and *in vivo* and *in vitro* biological activities of different parts of *C. maxima* was collected from published articles retrieved through several relevant databases including Google Scholar, PubMed, Chemical Abstract, Scifinder, Web of Science, and Scopus. The database was searched with the keywords such as *Citrus maxima,* pummelo, and *Citrus grandis* along with pharmacological activity, phytochemicals, ethnomedicinal uses, toxicity, etc.

## 3. Traditional Uses

It is well documented for its ethnomedicinal values in many countries [4, 5, 10, 11]. Fruits are used as stomach tonic, appetizer, cardiac stimulants and for the treatment of inflammation, cough, asthma, obesity, leprosy, mental aberration, epilepsy, headache, diarrhea [12–15], antipyretic, and antiemetics agents [16]. Pulp has been used traditionally for cosmetic purpose. The seeds are used against lumbago, dyspepsia, and coughs. Leaves are used for the treatment of epilepsy, cholera, and convulsive cough while decoction is useful on swellings and ulcers [17–19]. The details of traditional use of the plant are given in Table 2.

## 4. Bioactive Chemical Constituents

Phytochemicals belonging to different chemical classes such as alkaloids, saponins, carbohydrates, phenols, flavonoids, glycosides, anthraquinone, amino acids, carotenoids, and terpenoids are present [29–32].  Table 3 shows the details of phytoconstituents present, their classes, and plant parts used for isolation.

### 4.1. Alkaloids

Alkaloids have been isolated from most of the parts including stem, flower, fruit, peel, root, and bark of the plant. The structures of the isolated alkaloids are shown in Figure 2. Some of the isolated acridone alkaloids are citpressine-I and II*, 5*-hydroxynoracronycine, buntanine, citracridone-I, II, and III [35], citrusinine-I, grandisine-I and II, glycocitrine-I, natsucitrine-II, and prenylcitpressine [33, 34]. Alkaloids like buntanbismine, buntanmine A, afoline, baiyumine-A and -B, caffeine, citbismine-A, -B, and -C, citropone-A and -B, geibalansine, honyumine, pumiline, *p*-synephrine, theobromine, theophylline, and paraxanthine are also reported from the plant [28, 35, 37–39, 41, 43, 49].

### 4.2. Benzenoids

Benzenoids are the major volatile phytochemicals that are essential for attracting insects for pollination [70]. Some of the isolated benzenoids (Figure 3) are crenulatin, diphenylamine, methyl *N*-methyl anthranilate, and *p*-hydroquinone [34].

### 4.3. Coumarins

Different coumarins isolated from *C. maxima* are 5-methoxyseselin [49], 5-[(6′,7′-dihydroxy-3′,7′-dimethyl-2-octenyl)oxy]psoralen, 5-[(7′,8′-dihydroxy-3′,8′-dimethyl-2-nonadienyl)oxy]psoralen [50], 5-geranoxy-7-methoxy-coumarin [21], 5-demethyltoddannol, umbelliferone [33], 8-(3-hydroxy-2,2-dimethylpropyl)-7-methoxy-2H-chromen-2-one, auraptene [50], bergamottin, buntansin, citrubuntin [33], columbianoside I and II [51], crenulatin [33], epoxybergamottin [50], honyudisin, marmin, meranzin hydrate I, II, III, IV, paniculin III, scopoletin, suberenone, suberosin, ulopterol, umbelliferone, xanthoxyletin, and xanthyletin [33, 52]. Structures of some of these compounds are given in Figure 4.

### 4.4. Carotenoids

Carotenoids are important dietary constituents and also improve the immune response in the plant [71]. The isolated carotenoids from the fruit include *β*-carotene, phytoene, lutein, zeaxanthin, *α*-carotene, *β*-cryptoxanthin, and lycopene [45–48, 72].

### 4.5. Flavonoids

Flavonoids are one of the most reported chemical classes from this plant (Table 3). Apart from hesperidin, naringenin, and neohesperin, which are common in citrus plants, flavonoids like acacetin, apigenin, cosmosiin, diosmetin, diosmin, eriocitrin, hesperidin, honyucitrin, luteolin, isosinensetin along with polymethoxyflavones like 5,6,7,8,4′-(tangeritin or ponkanetin), 5,6,7,8,3′,4′-pentamethoxy-(nobiletin), and 5,7,4′-trimethoxy-(apigenin trimethyl ether) are also reported [62–65, 67]. Structures of some of the main flavonoids are shown in Figure 5.

### 4.6. Phenolics

Phenolics are essential phytochemicals against stress in plants [73]. Some of the isolated phenolic compounds (Figure 6) from its fruit are caffeic acid, 4-hydroxy-3-methoxy cinnamic acid, 4-hydroxycinnamic acid, gallic acid, and vanillic acid [59, 66].

### 4.7. Steroids

Some steroids including *β*-sitosterol, campesterol, daucosterol, and stigmasterol are reported from the peel, root, and fruit of this plant [21, 65, 68].

### 4.8. Terpenoids

*C. maxima* is also enriched with terpenoids. Triterpenoids like limonin, deacetynomilin, nomilin glucoside, deoxylimonin, obacunone glucosides, obacunone, and nomilinic acid are the major terpenoids (Figure 7) [28].

### 4.9. Carbohydrates and Amino Acids

Fructose, glucose, pectin, and sucrose are the different carbohydrates found in fruit, peel, and *C. maxima* leaves [29, 30]. Similarly, amino acids like aspartic acid, proline, alanine, glycine, serine, arginine, asparagine, lysine, glutamic acid, isoleucine, leucine, tryptophan were also isolated from *C. maxima* [29, 74].

### 4.10. Essential Oil Constituents

Essential oils are also recorded from its leaves, flower, and peel which includes (Z)-ocimene, 4-methyl-1-hexene, 3,3-dimethyl-1-hexene, geraniol, [75–77] geranyl acetate, limonene, geranyl formate, linalool, nerol, nerolidol, sabinene, *α, β* -pinene, *β-*farnesene, and *β*-myrcene [53, 55, 78].

### 4.11. Miscellaneous Compounds

In addition to the compounds mentioned above, a few compounds like L-ascorbic acid, citric acid, decyl acetate, fumaric acid, hexanal, malonic acid, succinic acid, *α-*tocopherol, pentadecanoic acid, hexadecanoic acid, tetradecanoic acid have been isolated from fruit juice, peel, and leaves of *C. maxima* [28, 79].

## 5. Pharmacological Activities

Various studies have been performed regarding the pharmacological effects of *C. maxima* extracts and their isolated compounds. Modern pharmacological studies confirm the traditional efficacy of this plant as an antiepileptic, antidepressant, and anti-inflammatory agent. The plant is highly potent for treating anxiety, depression, Alzheimer's disease (AD), and other neurological diseases. The plant also exhibits additional antioxidant, analgesic, hepatoprotective, antimicrobial, and anticancer activities. In this review, we collected the available information and described major pharmacological properties like antioxidant, antidepressant, anxiolytic, anti-Alzheimer's disease, antitumor, insecticidal, antidiabetic, antimicrobial, hepatoprotective, anti-obesity, anti-inflammatory, and analgesic activities.

### 5.1. Antioxidant Activity

Dulay et al. studied the antioxidant activity of leaf extracts of *C. maxima* along with two other plants, i.e., *C. microcarpa*, and *C. aurantium* by 2,2-diphenyl-1-picrylhydrazyl (DPPH) scavenging assay where *C*. *microcarpa* showed the highest scavenging activity of 48.67% followed by *C. maxima* having 43.51%, and *C. aurantium* had the lowest antioxidant capacity [80]. Fidrianny et al. also reported the antioxidant activity of its leaves, peel, and cortex extracts by DPPH and phosphomolybdenum assays. Data showed that the ethyl acetate extract of cortex exhibited the lowest IC_50_ value of 0.68 *μ*g/mL in DPPH scavenging activity, while ethyl acetate leaf extracts exhibited an IC_50_ value of 101.36 *μ*g/mL in the phosphomolybdenum assay [81].

The *in vivo* antioxidant activity of methanolic leaf extract (200 and 400 mg/kg, b.w.) was evaluated against paracetamol-induced hepatotoxicity in Wistar albino rats. Leaf extract at 400 mg/kg· b.w. showed reduced lipid peroxidation in paracetamol-treated rat liver as compared to that of saline control. It was also able to restore the depleted catalase and reduce glutathione levels in the paracetamol-intoxicated rat liver to the normal levels, indicating the *in vivo* antioxidant potential of extracts in paracetamol challenged rats [82]. The freeze-dried fruit extract of *C. maxima* exhibited 6609 *μ*·mol Fe^2+^/L antioxidant power through the ferric-reducing antioxidant powder (FRAP) assay which is very similar to the standard drug ascorbic acid [83]. The presence of major phytochemicals might be the reason for showing significant antioxidant activity by *C. maxima* extracts [14, 84, 85].

### 5.2. Antidepressant Activity

The aqueous leaf extracts (100, 200, and 300 mg/kg) of *C. maxima* were evaluated in mice for their antidepressant potential using different models. Fluoxetine (20 mg/kg, i.p.) and imipramine (30 mg/kg, i.p.) were used as standard drugs. The aqueous leaf extracts reduced the immobility time in both the tail suspension test (TST) and the forced swimming test (FST). The exact mechanism for exhibiting antidepressants was not reported, but it might be due to enhancement of norepinephrine neurotransmission in mice [20]. Similarly, the per-oral administration of ethanolic extracts (200 and 400 mg/kg) of *C. maxima* in mice increased the number of rearing in both the TST and FST models while imipramine (1 mg/kg) noticeably reduced the immobility time [86].

Hesperidin and naringin were evaluated against antidepressant activity using the FST and TST models. Both compounds exhibited significant antidepressant activity [87, 88]. The antidepressant effects of plant extracts might be due to the interaction with the serotonergic 5-HT1A and *κ*-opioid receptors [89, 90]. It was concluded that *C. maxima* extract was useful in its motor-stimulating effects.

### 5.3. Anti-Alzheimer's Disease Activity

Alzheimer's disease is a neurodegenerative progressive disease that occurs in the elderly population. During the experiments performed using Ellman's colorimetric and scopolamine-induced Alzheimer's methods, ethanolic, hexane, ethyl acetate, and aqueous extracts of *C. maxima* fruit peel exhibited potent anti-Alzheimer's activity. Similarly, it was found that the brain acetylcholinesterase level was decreased by leaf extract and showed anti-Alzheimer's activity [14, 90].

Naringin (40 and 80 mg/kg, p.o.) showed anti-Alzheimer's activity in colchicine tempted cognitive impaired rats through the elevated plus maze and Morris water mazemethods. Colchicine (15 *µ*g/5 mL) was given intracerebroventricularly which causes poor memory retention and reduces acetylcholinesterase activity in both the models [88]. The anti-Alzheimer's activity might be due to the development in the cognitive act and diminished oxidative stress by lowering malondialdehyde and nitrite levels. Also, it might be due to the renewal of superoxide dismutase, catalase, and glutathione S-transferase, and a reduction in glutathione as well as the acetylcholinesterase level in tested mice [91].

### 5.4. Anticancer and Antitumor Activity

The leaf extract of *C. maxima* tested against Ehrlich ascites carcinoma (EAC) models in swiss albino rats decreased the white blood cell (WBC) count and increased the lifespan. The biochemical parameters were also in the normal level as compared to the control group [92]. The methanolic extract of the leaves and its fractions in n-hexane, n-butanol, chloroform, ethyl acetate, and water were tested in normal cells and different cancerous cells through 3-(4,5-dimethylthiazol-2-yl)-2,5-diphenyl-tetrazolium (MTT) assay. Importantly, the chloroform fraction of leaf extract reduced the survival of HeLa cells [93].

Naringin exhibited potent anticancer activity in various experiments. Naringin (10, 25, and 35 mg/kg i.p.), when treated on rats bearing Walker 256 carcinosarcoma (W256) reduced tumor growth by 75% and TNF-*α* and IL-6 levels decreased in comparison with the control [94, 95]. Naringenin also exhibited cell proliferation and cell migration in B16F10 murine and SK-MEL-28 human melanoma cells. Hesperidin exhibited chemopreventive effects against an azoxymethane (AOM) induced carcinogenesis in the mouse colon. It was found to have significant reducing power for the multiplicities of AOM-induced aberrant crypt foci (ACF) and tumor incidence. It also decreased the proliferative marker proliferating cell nuclear antigen (PCNA) against AOM-induced colon carcinogenesis [96, 97]. The presence of flavonoids, limonoids, alkaloids, tannins, saponin, and bioflavonoids plays a prominent role in cancer prevention [59, 92, 98].

The anticancer activity of naringenin loaded liquid crystalline nanoparticles (LCNs) was evaluated against human lung epithelial carcinoma (A549) and airway epithelium derived basal cells (BCi-NS1.1). Mainly antiproliferative, antimigratory, and anticolony formation activity were studied in which naringenin LCNs showed its significant anticancer properties by inhibiting the migratory and proliferation properties of cells [99].

### 5.5. Antidiabetic Activity

The *in vitro* enzyme inhibitory activity of *C. maxima* fruit juice was examined against *α*-glucosidase and *α*-amylase. The percentage inhibition by fruit juice for *α*-amylase was 75.55%–79.75% and, for *α*-glucosidase, it was 70.68%–72.83% [100]. The hypoglycaemic property of fruit juice was examined in the streptozotocin (STZ)-induced diabetes mellitus model. The glucose level was lowered in experimental rats than in control rats which is due to the peripheral utilization of glucose or inhibition of gluconeogenic enzymes [23].

The antidiabetic activity of the leaf extracts (200 and 400 mg/kg, b.w.) was evaluated in STZ (65 mg/kg) induced diabetic rats using glibenclamide (0.5 mg/kg, p.o) as the reference standard. The blood glucose level and serum biochemical parameters were measured and found to be normalized in experimental rats than in the control group [101]. The antidiabetic effect of neohesperidin on *α*-amylase and *α*-glucosidase improved postprandial hyperglycemic conditions [102]. The antioxidant activity of plants may lead to their defensive effects against chronic metabolic disorders [103].

The antidiabetic activity of methanolic and ethanolic leaf extracts (100 and 200 mg/kg of each extract) of *C. maxima* was also evaluated against the alloxan (90 mg/kg b.w.) induced diabetes model in mice while glibenclamide (5 mg/kg, p.o.) was used as the standard. The plasma glucose level and parameters of serum lipid profile, serum glutamic pyruvic transaminase (SGPT), serum glutamic oxaloacetic transaminase (SGOT), and C-reactive protein (CRP) were measured and found to be inhibited by the leaf extract in experimental mice as compared to control mice. This finding suggests that both extracts have significant hypoglycaemic effects and can ameliorate the altered lipid profile in diabetic mice. Moreover, the results suggested that the extracts of *C. maxima* leaf can restore altered levels of liver function enzymes and CRP in diabetic mice, highlighting the hepatoprotective and cardioprotective potentiality of this plant [104].

### 5.6. Antimicrobial Activity

The antibacterial activity of *C. maxima* has been widely studied. The ethanolic leaf extract exhibited antibacterial activity against *Pseudomonas aeruginosa* and *Escherichia coli* [17]. The ethanolic pulp and seed extracts also exhibited antibacterial activity against *Bacillus subtilis, Staphylococcus aureus*, and *Escherichia coli* in the disc diffusion method [105]. In another study, the methanolic extracts of the leaves, seeds, fruits peel, and barks were tested against *Escherichia coli*, *Klebsiella pneumonia*, and *Staphylococcus aureus*. Pulp extract showed the highest zone of inhibition (ZOI) of 26 mm in *Klebsiella pneumonia,* while none of the other extracts showed significant ZOI. The aqueous extract of the pulp also showed highest antibacterial activity (ZOI of 27 mm) against *Staphylococcus aureus* [106]. The presence of naringenin and hesperidin might be responsible for its antibacterial activity. The antibacterial activity of hesperidin against Gram-positive and Gram-negative bacteria has already been established [107]. The essential oils from *C. maxima* also demonstrated antibacterial activity against *Escherichia coli*, *Bacillus subtilis*, *Staphylococcus aureus*, *Pseudomonas aeruginosa*, *Bacillus licheniformis*, and *Bacillus altitudinis* in the broth dilution method [108].

The significant antifungal activity of ethanolic and aqueous leaf extracts against *Fusarium moniliforme*, *Aspergillus niger*, and *Mucor plumbeus* fungus was reported by Hemalatha through the agar-well diffusion and disc diffusion methods [109]. Similarly, Jing et al. reported that limonene is effective against *Aspergillus niger, A. flavus, A. fumigatus, A. terreus, A. parasiticus, Penicillium chrysogenum, P. digitatum, P. italicum, P. expansum, Fusarium oxysporum, F. proliferatum,* and *Alternaria alternata* [110].

### 5.7. Hepatoprotective Activity

*C. maxima* leaf and peel extracts revealed liver protective effect in carbon tetrachloride-induced hepatotoxicity in Wistar rats. Significant reduction of aspartate aminotransferase (AST), alanine transaminase (ALT), and alkaline phosphatase (ALP) levels in experimental rats proved its hepatoprotective activity [111, 112]. In another study, hepatoprotective effects of *C. maxima* methanolic leaf extract (200 mg/kg, b.w.) was examined in paracetamol-induced hepatotoxicity in rats. In this study, leaf extracts were administered for 7 days, paracetamol (2 g/kg) was administered at 5^th^ day, and silymarin (100 mg/kg, b.w.) was used as the standard drug. Liver was extracted and liver function markers, total bilirubin, total protein in blood serums, and hepatic antioxidants in liver homogenate were evaluated and found normal as compared to the control group [113]. Leaf extracts having antioxidant property might be responsible to decrease the distortion of hepatocytes by elevating the hepatic antioxidant enzymes levels [31].

### 5.8. Anti-obesity Activity

The anti-obesity activity of ethanolic leaf extract (200 and 400 mg/kg) against olanzapine-induced obesity and cafeteria diet-induced obesity in rats. Body weight, body temperature, and serum parameters were evaluated and found significantly decreased in their values as compared to the obese control group [114]. Ding et al. fed the *C. maxima* ethanolic peel extract to the mice along with Chow diet for 8 weeks. The diet lowered the weight, decreased fasting blood glucose levels, and also reduced liver lipid and serum insulin levels [115]. Hesperidin also regulates the lipid and glucose metabolism and indirectly facilitates NF-*κ*B signalling way to control inflammation which helps in controlling obesity [116, 117].

### 5.9. Analgesic and Anti-Inflammatory Activity

Various parts of *C. maxima* have shown analgesic and anti-inflammatory properties. The analgesic property of the methanolic extract of its peel was examined by formalin-induced licking and biting model and acetic acid-induced writhing model. The extract at a higher dose (500 mg/kg) showed satisfactory analgesic activity (73.34%) in the acetic acid-induced pain model as compared to 87.13% activity shown by standard drug diclofenac sodium at 10 mg/kg dose [118]. In another experiment, the analgesic activity of leaf, stem, and fruit was compared by using the tail-flick method in rats, acetic acid-induced writhing, and the hot plate method in mice. Results showed that the leaf extract at 300 mg/kg showed significant analgesic activity in all the models used [119]. Similarly, Kundusen et al. also showed its anti-inflammatory activity in rats when evaluated using formalin, carrageenan, and dextran-induced acute rat paw edema models. Many studies suggested that the mechanism responsible for analgesic and anti-inflammatory activity is due to inhibition of prostaglandin synthesis. Also the presence of flavonoids and their respective aglycones like hesperetin and naringenin might be the reason for the potent anti-inflammatory and analgesic activity [10, 118–120].

### 5.10. Other Uses

*C. maxima* fruits are known for their characteristic flavor, making them suitable for breakfast. The peel oil is used as a flavoring agent in food, pharmaceutical products, cosmetics, and perfumery items [25]. Due to refreshing and good-smelling properties, its essential oils are also added in toiletry and insecticidal products [121]. The pectin in rind is used in making jellies and candies, and wood can be used for making suitable tool handles [122].

## 6. Conclusion and Future Prospects

*C. maxima* offers a wide range of medicinal and nutritional uses. Almost all parts of the plant, including whole fruit, fruit pulp, fruit rind, fruit peel, juice, flower, leaf, seed, and essential oils, are traditionally used for the treatment of various diseases. A phytochemical profile showed the presence of many bioactive chemical constituents under several chemical classes including alkaloids, benzenoids, coumarins, carotenoids, phenols, flavonoids, tannin, terpenoids, saponins, amino acids, and carbohydrates. Extracts of various plant parts showed numerous pharmacological properties like antioxidant, antimicrobial, analgesic, anticancer, antidiabetics, anti-inflammatory, anti-Alzheimer's, insecticidal, anxiolytic, hepatoprotective, antimalarial, and anti-obesity activities. Isolated compounds like hesperidin, limonene, naringenin, naringin, and neohesperidin have been reported to possess bioactivities like antioxidant, antidepressant, antitumor, anticancer, antimicrobial, hepatoprotective, anti-obesity, insecticidal, analgesic activity, anxiolytic, anti-Alzheimer, antiulcer, and antidiabetic activities. The essential oils from fruits and leaves have enhanced their use in the perfumery and cosmeceutical industry.

Despite the tremendous ethnomedicinal reports, preliminary studies, and promising results, correlations between traditional uses and pharmacological activities are still needed to be established. Bioassay-guided fractionation and isolation of compounds is needed to find more potent and novel compounds for the discovery of lead compounds and to demonstrate their molecular mechanisms to design effective herbal products and functional foods. Extensive *in vivo* pharmacological tests, pharmacokinetic studies, clinical trials, and toxicity studies are needed. The information regarding the therapeutic dose, dosage form, and safety of the plant products is still an area to be explored. Since the plants can easily grow in south-east Asia including Nepal and India, local farmers can be promoted for the mass cultivation of this plant and small-scale herbal pharmaceutical and juice industries can be established. Thus, viable products and food supplements of this plant species can be designed and marketed at an international level which will ultimately uplift the economic status of the local producer.

## Figures and Tables

**Figure 1:** Photographs of tree (a), ripe fruits (b), fruit (c), fruit internal section (d), the flesh (e), and seeds (f) of *C. maxima*.

**Figure 2:** Chemical structures of some alkaloids from *C. maxima*.

**Figure 3:** Chemical structures of some benzenoids from *C. maxima*.

**Figure 4:** Chemical structures of some coumarins from *C. maxima*.

**Figure 5:** Chemical structures of some flavonoids from *C. maxima*.

**Figure 6:** Chemical structures of phenolic acids from *C. maxima*.

**Figure 7:** Chemical structures of some terpenoids from *C. maxima*.

**Table 1:** Some common names of *Citrus maxima*.

Language	Common name
Nepali	Bhogate
English	Pummelo, shaddock, pumelo
Sanskrit	Madhukarkati
Italian	Pompelmo
French	Pamplemousse
Portuguese	Jamboa
Spanish	Pamelmusa
Polish	Pompela
Indonesian	Jeruk Besar, Jerukbali

**Table 2:** Traditional uses of different parts of *Citrus maxima* in different countries.

Parts	Ailments and mode of application	Areas	References
Essential oil	Sedative in nervous affections, convulsive cough, haemorrhagic diseases, and epilepsy	India	[20]
Fruits pulp	Pulp juice as antitoxic, appetizer, cardiac stimulant, and stomach tonic	Mediterranean region	[21]
Fruits rind	Antiasthmatic, brain tonic, antiemetics, griping in the abdomen, diarrhea, and headache	India	[7]
Fruits	The juice is applied to pimples and dandruff	Nepal	[22]
Fruits	Leprosy, asthma, cough, hiccough, mental aberration, and epilepsy	India	[7]
Fruits	Diabetes	Nigeria	[23]
Fruits	Headache, flu, fever, sore throats, breathing disorders, and dyspepsia	Thailand	[24]
Fruits peel	A decoction of peel has been used to improve coughs, swellings, ulcers, and epilepsy	Kenya	[25]
Fruits peel	Obesity and hypertension	China	[26]
Leaves	Leaves are chewed to expel the intestinal worms	Nepal	[22]
Leaves and flowers	As sedative in nervous affections, convulsive cough, cholera, epilepsy, haemorrhagic diseases, and a lotion of boiled leaves used in painful swellings	India	[27]
Leaves, flowers, fruits, and seed	As decoctions to treat coughs, fevers, and gastric disorders	The Philippines and southeast Asia	[28]

**Table 3:** Details of phytochemicals present in *Citrus maxima*.

Class	Compounds name	Plant parts used	References
Acridone alkaloids	5-Hydroxynoracronycine	Stem bark	[33]
	Buntanine	Root bark	[34]
	Citpressine-I, II	Stem bark and root bark	[33, 34]
	Citracridone-I, II	Stem bark and root bark	[33, 34]
	Citracridone-III	Stem bark	[35]
	Citrusinine-I	Stem bark	[33]
	Glycocitrine-I	Stem bark	[35]
	Grandisine-I and II	Stem bark	[35]
	Grandisinine	Stem bark	[33]
	Natsucitrine-II	Stem bark	[35]
	Prenylcitpressine	Stem bark	[33]
	Atalafoline	Stem bark	[28]
	Baiyumines A, B	Root bark	[36]
	Buntanbismine	Stem bark	[37]
	Buntanamine-A	Stem bark	[33]
	Caffeine	Flower	[38]
	Citbismines A, B, C	Root	[39]
	Citropone-A and -B	Root bark	[40]
	Geibalansine	Stem bark	[28, 41]
	Honyumine	Root bark	[42]
	Pumiline	Root	[4]
	p-Synephrine	Fruits and leaves	[43]
	Theobromine	Flower	[38]
	Theophylline	Flower	[38]
	Paraxanthine	Flowers	[38]

Benzenoids	Diphenylamine	Root bark, stem bark, fruit juice	[34]
	Methyl N-methylanthranilate	Leaves	[44]
	p-Hydroquinone	Root bark, stem bark, fruit juice	[34]

Carotenoids	Phytoene	Fruits	[45–47]
	*α*-carotene	Fruits	[45–47]
	*β*-carotene	Fruits	[45–47]
	*β*-cryptoxanthin	Fruits	[45–47]
	Lutein	Fruits	[48]
	Zeaxanthin	Fruits	[48]
	Lycopene	Fruits	[48]

Coumarins	5-Methoxyseselin	Root bark	[49]
	5-[(6′,7′-Dihydroxy-3′,7′-dimethyl-2-octenyl)oxy] psoralen	Fruit peel	[50]
	5-[(7′,8′-Dihydroxy-3′,8′-dimethyl-2-nonadienyl)oxy] psoralen	Fruit peel	[50]
	5-Geranoxy-7-methoxy-coumarin	Root and stem bark	[21]
	5-Demethyltoddannol	Stem bark	[33]
	Umbelliferone	Stem bark	[33]
	8-(3-Hydroxy-2,2-dimethylpropyl)-7-methoxy-2*H*-chromen-2-one	Fruit peel	[50]
	Auraptene	Peel	[50]
	Bergamottin	Peel	[33]
	Buntansin	Stem bark	[33]
	Citrubuntin	Stem bark	[33]
	Columbianosides I, II	Fruit pericarp	[51]
	Crenulatin	Stem bark	[33]
	Epoxybergamottin	Peel	[50]
	Honyudisin	Stem bark	[34]
	Marmin	Peel	[50]
	Meranzin hydrate I, II, III, IV	Fruit pericarp	[51]
	Paniculin III	Fruit pericarp	[51]
	Scopoletin	Stem bark	[33]
	Suberenone	Stem bark	[33]
	Suberosin	Stem bark	[33]
	Ulopterol	Stem bark	[33]
	Umbelliferone	Fruit flesh, stem bark	[33, 52]
	Xanthoxyletin	Stem bark	[33]
	Xanthyletin	Stem bark	[33]

Constituents in essential oil (volatile constituents)	(*Z*)-Ocimene	Flower, peel, leaves	[53]
	4-Methyl-1-hexene	Flower, peel, leaves	[54]
	3,3-Dimethyl-1-hexene	Flower, peel, leaves	[54]
	Geraniol	Flower, leaves	[55, 56]
	Geranyl formate	Flower, peel, leaves	[54]
	Geranyl acetate	Flower, peel, leaves	[54]
	Limonene	Flower, peel, leaves	[53]
	Linalool	Flower, peel, leaves	[53]
	Nerol	Fruit peel	[57]
	Nerolidol		
	Sabinene	Fruit peel	[53, 55]
	*α, β*-Pinene	Flower, peel, leaves	[53–55]
	*β-*Farnesene	Flower	[56]
	*β*-Myrcene	Flower, leaves	[53]

Flavonoids	Acacetin	Leaves	[58]
	Apigenin	Fruit	[59]
	Cosmosiin	Leaves	[28, 58]
	Diosmetin	Flavedo	[58]
	Diosmin	Flavedo, fruit juice	[58]
	Eriocitrin	Albedo	[58]
	Hesperidin	Peel, fruit juice	[60]
	Honyucitrin	Root bark	[58]
	Isosinensetin	Peel	[58]
	Luteolin	Fruit juice, leaves, peel	[58]
	Naringenin	Fruits peel	[61, 62]
	Naringin	Fruits peel	[61–65]
	Naringin 4′-glucoside	Flavedo, albedo	[28, 58]
	Narirutin	Fruit juice, peel, leaves	[60]
	Neodiosmin	Fruit juice, peel	[28, 58]
	Neoeriocitrin	Fruit juice, peel, leaves	[58]
	Neohesperidin	Fruit juice, peel, leaves	[60]
	Neoponcirin	Fruit juice, peel	[66]
	Nobiletin	Peel	[58]
	Poncirin	Albedo, leaves	[66]
	Quercetin	Fruit juice	[28, 58]
	Rutin	Peel, leaves	[58]
	Tangeretin	Fruit peel	[67]
	Nobiletin	Fruit peel	[67]
	Apigenin trimethyl ether	Fruit peel	[67]
	Sinensetin	Fruit peel	[67]
	5,7,3′,4′-Tetramethoxyflavone	Fruit peel	[67]
	5,7,8,3′,4′-Penta-methoxyflavone	Fruit peel	[67]

Phenolics	Ferulic acid	Fruit	[59]
	4-Hydroxycinnamic acid	Fruit	[59]
	Caffeic acid	Seed	[28]
	Gallic acid	Fruit	[59, 66]
	Vanillic acid	Fruit	[59]

Steroids	*β*-Sitosterol	Peel, root, fruit	[21, 65, 68]
	Campesterol	Peel, root	[21, 68]
	Daucosterol	Peel, root	[21, 68]
	Stigmasterol	Peel, root	[21, 68]

Triterpenes	Deacetynomilin	Seed	[28]
	Deoxylimonin	Seed, fruit, pulp	[28]
	Limonin	Seeds, fruit, peel, leaves	[69]
	Nomilin glucoside	Peel	[28]
	Nomilinic acid	Seed	[28]
	Obacunone	Leaves, seed, fruit pulp	[28]
	Obacunone glucoside	Seed	[28]

## Data Availability

No new experimental data were generated during the preparation of this review article.

## Abbreviations

ABTS: 2,2′-Azino-bis (3-ethylbenzothiazoline-6-sulfonic acid)
AD: Alzheimer's disease
ALP: Alkaline phosphatase
ALT: Alanine transaminase
AST: Aspartate amino transferase
COX-2: Cyclooxygenase-2
EAC: Ehrlich ascites carcinoma
EPM: Elevated plus maze test
FST: Forced swimming test
HDL: High-density lipoproteins
HUVEC: Human umbilical vein endothelial cell
IL-6: Interleukin 6
iNOS: Inducible nitric oxide synthase
LDL: Low-density lipoproteins
MIC: Minimum inhibitory concentration
MTT: 3-(4,5-Dimethylthiazol-2-yl)-2,5-diphenyl-tetrazolium
PPARs: Peroxisome proliferator-activated receptors
SGOT: Serum glutamic oxaloacetic transaminase
SGPT: Serum glutamic pyruvic transaminase
TNF-*α*: Tumor necrosis factor-alpha
ZOI: Zone of inhibition.
DPPH: 2,2-diphenyl-1-picrylhydrazyl
TST: Tail suspension test
